# Effect of Intraarticular Injection of Platelet-Rich Plasma on Knee Osteoarthritis: A Multicenter Retrospective Clinical Study

This article has been retracted.

**DOI:** 10.1155/2022/1788153

**Published:** 2022-01-07

**Authors:** Bin Zhang, Jiasheng Yu, Daobo Fan, Lei Bao, Dongqian Feng

**Affiliations:** Department of Orthopedics, Shuyang Hospital Affiliated to Yangzhou University School of Medicine (Shuyang Hospital of Traditional Chinese Medicine), No. 28 Shanghai Middle Road, Shuyang, Suqian, Jiangsu, China

## Abstract

This study aimed to evaluate the effect of intraarticular injection with platelet-rich plasma on knee osteoarthritis. A total of 250 patients with stages I–III osteoarthritis from December 2018 to June 2020 were included in this study. All the patients had received autologous PRP injection (3 ml) into the affected knee joint every week for totally 3 injections. The VAS score and WOMAC index were used to evaluate knee function before and at 3 days, 1 month, and 3 months after injection. A total of 250 patients were enrolled in this study, including 130 patients in the PRP group and 120 patients in the control group. The content of platelets in PRP of patients in the PRP group was 958.0 ± 283.1 × 10^9^/L. The VAS score and WOMAC index of patients in the PRP group before treatment were not significantly different from those in the control group. At 3 days, 1 month, and 3 months after PRP treatment, the VAS score and WOMAC index of the PRP group were significantly lower than those of the control group. PRP is effective in treatment of knee osteoarthritis. The pain symptoms can be alleviated at 3 days after injection.

## 1. Introduction

Knee osteoarthritis is one of the common degenerative diseases in the clinic, especially in people aged more than 65 years and with a high amount of exercise [1]. High amount of exercise is an important factor of KOA in Chian. Nonsteroidal anti-inflammatory drugs, chondroitin sulfate, glucosamine, hyaluronic acid, and glucocorticoids are currently the main conservative treatments for this disease [2]. However, the above methods have different degrees of adverse reactions, and the cartilage tissue healing ability is poor, so it can only achieve short-term analgesic and anti-inflammatory effects, and the long-term clinical effect is not good. Platelet-rich plasma (PRP) is a concentrated polymer with a higher concentration of platelets obtained after autologous blood concentration. The platelet concentration is 3–5 times higher than normal blood. PRP contains high concentrations of self-derived growth factors, including the vascular endothelial growth factor, platelet-derived growth factor, and transforming growth factor *β*, which promote the proliferation of chondrocytes and the synthesis of extracellular matrix [3–5]. As well known, PRP and MSCs are the hotspots of biological engineering research worldwide. In addition, PRP is easy to prepare, relatively low cost, and high in safety, so it is increasingly used in the field of sports system injuries. At present, there have been clinical studies on the treatment of osteoarthritis by PRP injection, but the curative effect is not consistent. The possible reason is that the difference in the preparation method results in a large difference in the cellular components of PRP [6].

This study intends to observe the early clinical efficacy of leukocyte-removed PRP in the treatment of osteoarthritis and to provide reference for clinical PRP in the treatment of knee osteoarthritis. This study is a multicenter clinical study and included patients from three clinical medical centers. The sample size of this study is larger than that of previous studies.

## 2. Methods

### 2.1. Patients

This study included 250 patients with knee osteoarthritis admitted to three medical centers from December 2018 to June 2020. It is planned to include 130 patients as the PRP treatment group and 120 patients as the control group. The inclusion criteria of this study are as follows: (1) knee joint swelling or pain (≥4 months), (2) knee joint degeneration confirmed by imaging (X-ray or MRI), and (3) Kellgren-Lawrence grades I–III. Exclusion criteria of this study are as follows: (1) age> 70 years, (2) Kellgren-Lawrence classification > grade III, knee varus or valgus> 5°, (3) infection, rheumatoid arthritis, diabetes, and severe ischemic heart disease, (4) complicated with hematological diseases or hemoglobin <11 g/L, platelets <1.5 × 10^9^/L, (5) have taken nonsteroidal anti-inflammatory drugs (NSAIDs), anticoagulants, or antiplatelet drugs within 1 week, and (6) pregnant women and breastfeeding women.

### 2.2. PRP

All patients completed relevant examinations and collected the patient's own platelets using the XCF3000 blood component separator. The blood flow rate was 60 ml/min, the collection time was 20–30 min, and the total circulation volume was 400–550 ml. A total of 15–20 ml platelet-rich plasma was collected. Reserve about 2 ml of PRP for cytological determination and the remaining PRP for injection into the knee joint cavity.

The patient lies on his back, exposing the knee joint, and the affected knee joint is slightly flexed. Routine disinfection is done with iodophor. Take the needle point into the patellofemoral joint space at the outer edge of the patella and puncture the knee joint cavity with a 21G needle. If there is effusion, first draw out the effusion in the knee joint, then inject PRP, and inject 3 ml on each knee joint. Sterile excipients cover the puncture point after injection. Slightly bend and extend the knee joint several times to make the PRP fully cover the articular surface. After the injection, the patient is instructed to avoid strenuous exercise, and the puncture point should be kept away from water within 1 day. The injection was once every 1 week for a total of 3 consecutive injections. Avoid using nonsteroidal anti-inflammatory drugs during treatment and within 1 week after treatment.

### 2.3. Data Recording

We recorded the adverse events, treatment methods, and treatment results after blood sampling and knee joint injection. The visual analogue scale (VAS) score and Western Ontario and McMaster Universities Osteoarthritis Index (WOMAC) index were used for evaluation before injection and 3 days, 1 month, and 3 months after injection. We compared the evaluation results at various time points before and after treatment. Among them, the higher the VAS score, the more severe the pain, and the higher the WOMAC index, the more severe the knee osteoarthritis.

### 2.4. Statistical Analysis

Statistical analysis was performed by Statistical Package for Social Science (SPSS version 25.0, Armonk, NY, USA) and R (version 4.0.5). Continuous variables were expressed in mean ± standard deviation or median (interquartile range (IQR)) as appropriate. Differences between subgroups were analyzed using the *χ*^2^ or Fisher's exact test for categorical parameters and Student's *t*-test or Mann–Whitney's test for continuous parameters as appropriate. All statistical tests were 2-sided. Statistical significance was taken as *P* < 0.05.

## 3. Results

### 3.1. Patients

A total of 250 patients were enrolled in this study, including 130 patients in the PRP group and 120 patients in the control group. The baseline conditions of the two groups of patients are given in Table 1. The sex ratios of the two groups of patients were similar, and the ages of the two groups were not much different. There was no statistically significant difference in the complete blood count between the two groups. The content of platelets in PRP of patients in the PRP group was 958.0 ± 283.1 × 10^9^/L, and the counts of white blood cells and red blood cells in PRP were almost zero. There was no significant statistical difference in the results of biochemical examinations between the two groups of patients.

### 3.2. Complications

In the PRP patient group, 11 patients had transient dizziness during injection, and their symptoms were relieved after rest. Hypocalcemia was considered due to the effect of anticoagulants during platelet separation. Two patients developed swelling and pain in the lower limbs. Five patients were considered to be infected. No patient had other complications such as venous thrombosis of the lower extremities.

### 3.3. Effectiveness

The VAS score and WOMAC index of patients in the PRP group before treatment were not significantly different from those in the control group. At 3 days, 1 month, and 3 months after PRP treatment, the VAS score and WOMAC index of the PRP group were significantly lower than those of the control group (Table 2).

### 3.4. Analysis of Related Factors of VAS Score

We analyzed clinical variables related to the decline in VAS scores in the PRP patient group. There was no significant correlation between baseline variables such as the patient's gender and age and the patient's VAS score. The platelet count in PAP is correlated with the improvement of the patient's VAS score (Table 3).

## 4. Discussion

Knee osteoarthritis is a noninfectious joint inflammation characterized by progressive degeneration of knee cartilage and bone hyperplasia [7, 8]. Nonsurgical treatment methods mainly include oral nonsteroidal anti-inflammatory drugs, amino sugar-like articular cartilage nutrition drugs, and intraarticular injection of glucocorticoids and hyaluronic acid, but there are adverse digestive system reactions, chondrocyte toxicity, and immune reactions. Platelet-rich plasma is a platelet concentrate obtained after centrifugation of autologous whole blood and contains high concentrations of autologous source platelets and fibrinogen. Among them, growth factors released after activation of platelets can promote cell proliferation and release extracellular matrix, which helps repair cartilage damage, and is easy to prepare and safe to use. Therefore, PRP is increasingly used in the treatment of knee osteoarthritis [9].

The retrospective study of Sanchez et al. on patients with knee osteoarthritis showed that intraarticular injection of PRP was better than sodium hyaluronate injection in reducing knee joint pain and improving knee joint function. Kon et al. followed up 100 cases (115 knees in total) with PRP in the treatment of knee osteoarthritis. Compared with before the injection, 2 months after the injection, the patient's knee joint pain was reduced and the knee joint function score improved; but in the subsequent 12-month follow-up, the patient's pain score and knee joint score function gradually decreased. The author believes that intraarticular injection of PRP can help improve the pain symptoms and functional scores of patients with mild osteoarthritis. In this study, it was observed that after PRP injection treatment of knee osteoarthritis, the patient's symptoms were relieved, and joint function was relieved at the early stage (day 3) [10]. VAS scores and joint function scores at 3 days, 1 month, and 3 months after injection were significantly different from those before injection (*P* < 0.05).

The painful symptoms of knee osteoarthritis are related to the increase in the level of local inflammatory factors in the knee joint. In addition to promoting the growth of tissue cells, PRP also contains growth factors and inflammatory regulators to regulate inflammation. Zhang et al. observed the changes in the level of IL-17 in the synovial fluid of the knee joint cavity of 30 patients with osteoarthritis before and after PRP injection [11]. PRP injection can reduce the level of IL-17 in the knee joint cavity of the patient, reduce the patient's pain score, and improve the knee joint function. Zhang et al. observed the effect of growth factors in PRP on inflammatory factors in injured tendon tissue in mice [12, 13]. Studies have shown that the hepatocyte growth factor in PRP can reduce IL-1*β*-mediated COX-1, COX-2, and COX-1 in the inflammatory response, the level of mPGES-1 and other inflammatory factors. Van Buul et al. showed through in vitro experimental studies that PRP release can inhibit a series of inflammatory reactions caused by IL-1*β*, a common inflammatory factor in osteoarthritis [14, 15]. In this study, it was observed that the patient's pain was significantly reduced in the short-term (day 3) after injection of PRP, which may be related to the reduction of local inflammatory factors in the knee joint by PRP.

The production of platelet-rich plasma mainly uses the secondary centrifugation method, but in the separation process, in order to collect as many platelets as possible, a large number of white blood cells will be collected at the same time. This may be one of the reasons for the early joint swelling and increased pain after injection one. The platelet-rich plasma collected in this study adopts the separation and replacement method, which avoids the excessively high white blood cell concentration caused by the conventional centrifugation method. Follow-up patients did not observe obvious swelling or pain after injection, which may be related to low white blood cell concentration. The shortcomings of this study are that the sample size is small, the follow-up time is short, and the influence of the patient's body mass index is not considered. In future clinical studies, the number of samples should be further accumulated, and the follow-up time should be extended to provide stronger evidence for the choice of clinical treatment.

## 5. Conclusion

PRP is effective in treatment of knee osteoarthritis. The pain symptoms can be alleviated at 3 days after injection.

## Figures and Tables

**Table 1:** The baseline characteristics of the included patients.

Clinical parameters	PRP group, *N* = 130	Control group, *N* = 120	*P* value
Gender (N)			0.776
Male	80	75	
Female	50	55	
Age (years)	46.8 ± 15.7	51.2 ± 14.3	0.545
Knees involved (*N*)	48	56	0.876
Whole blood count (×10^9^/L)			
Platelet	243.6 ± 62.5	234.2 ± 42.3	0.453
WBC	6.0 ± 1.9	6.3 ± 1.4	0.478
RBC	4.5 ± 0.4	4.3 ± 0.3	0.674
PRP (×10^9^/L)			
Platelet	958.0 ± 283.1	—	—
WBC	0.0 ± 0.0	—	—
RBC	0.5 ± 0.2	—	—
ALT (IU/L)	24.0 ± 3.2	25.2 ± 3.5	0.786
AST (IU/L)	22.0 ± 1.7	22.7 ± 1.4	0.876
Albumin (g/L)	45.6 ± 12.4	47.1 ± 11.4	0.956
Total bilirubin (*μ*mol/L)	13.2 ± 1.3	15.1 ± 1.2	0.784
INR	0.8 ± 0.1	0.7 ± 0.2	0.554
Triglycerides (mmol/L)	1.0 ± 0.3	1.1 ± 0.2	0.675
Cholesterol (mmol/L)	4.1 ± 1.2	3.9 ± 1.1	0.778
HDL-C (mmol/L)	1.3 ± 0.3	1.2 ± 0.2	0.893
LDL-C (mmol/L)	2.4 ± 0.1	2.5 ± 0.2	0.934
Creatinine (*µ*mol/L)	77 ± 12	75 ± 9	0.757

**Table 2:** Comparison of the VAS score and WOMAC score in the PRP and control groups.

Time point		PRP group		Control group	
		VAS	WOMAC	VAS	WOMAC
T0	Preinjection	5.2 ± 1.8	30.8 ± 15.4	5.4 ± 1.4	31.7 ± 12.3
T1	3 days after injection	2.8 ± 1.3	14.9 ± 6.1	4.9 ± 1.5	28.3 ± 11.2
T2	1 month after injection	2.3 ± 1.3	14.5 ± 6.5	4.6 ± 1.2	29.3 ± 10.9
T3	3 months after injection	2.4 ± 1.2	13.9 ± 5.8	4.4 ± 1.6	27.3 ± 12.3

**Table 3:** Clinical factors associated with the VAS score in the PRP group.

Clinical parameters	OR (95% CI)	*P* value
Male (versus female)	1.12 (0.95–1.26)	0.089
Age (per year increase)	1.56 (0.69–2.47)	0.124
Knees involved	1.12 (0.89–1.42)	0.178
Platelet count^*∗*^	1.41 (0.78–1.98)	0.081
WBC count^*∗*^	1.21 (0.78–1.56)	0.074
RBC count^*∗*^	1.25 (0.56–1.79)	0.091
Platelet count^#^	1.56 (1.23–1.76)	0.012
WBC count^#^	—	—
RBC count^#^	—	—

^*∗*^Whole blood count. ^#^PRP.

## Data Availability

The simulation experiment data used to support the findings of this study are available from the corresponding author upon request.
